# Pregnancy and Venous Thromboembolism: Risk Factors, Trends, Management, and Mortality

**DOI:** 10.1155/2020/4071892

**Published:** 2020-04-11

**Authors:** Mohammed A. Alsheef, Alhanouf M. Alabbad, Rowida A. Albassam, Rawan M. Alarfaj, Abdul Rehman Z. Zaidi, Ohoud Al-Arfaj, Amani Abu-Shaheen

**Affiliations:** ^1^Medical Specialties Department, King Fahad Medical City, Riyadh, Saudi Arabia; ^2^College of Pharmacy, Princess Nourah bint Abdulrahman University, Riyadh, Saudi Arabia; ^3^Department of Clinical Pharmacy, King Fahad Medical City, Riyadh, Saudi Arabia; ^4^Department of Scientific Writing, Research Center, King Fahad Medical City, Riyadh, Saudi Arabia

## Abstract

**Background:**

Pregnancy is one of the major risk factors for the development of venous thromboembolism (VTE).

**Objective:**

To elucidate the circumstances surrounding pregnancy-induced deep vein thrombosis (DVT) and pulmonary embolism (PE), assess potential factors triggering thrombosis (e.g., thrombophilia, obesity, age, parity, and family history), initial and long-term management, and assess recurrence rate and mortality for VTE in pregnant Saudi women.

**Methods:**

A retrospective chart review of 180 patients with objectively confirmed VTE (DVT, PE, or both) that occurred during pregnancy, or the postpartum period was conducted. All patients who experienced episodes of objectively confirmed VTE were included.

**Results:**

Overall, 180 patients were included. Further, 60% (*n* = 109) and 40% (*n* = 71) of the VTE cases occurred during the postpartum and antenatal periods, respectively. Cesarean section was the most prevalent risk factor among study participants (*n* = 86 (47.8%)), followed by obesity (*n* = 73 (40.6%)). The most common clinical presentations were lower leg pain (57.2%) and lower limb swelling (54.4%). VTE recurrences were observed in approximately 11% of the participants, and maternal mortality occurred in 2 (1.1%) cases.

**Conclusion:**

Pregnancy was the most common provoking factor for VTE in our study. Pregnant women should undergo formal, written assessments of risk factors for VTE at the first visit and delivery. Larger studies with a randomized design, and control groups are required to confirm the current findings.

## 1. Introduction

Pregnancy is one of the major risk factors in the development of venous thromboembolism (VTE). The risks of VTE during pregnancy and the postpartum period are increased approximately five- and 60-fold, respectively [1].

The actual incidence of VTE among pregnant women may be overestimated if the diagnosis is based on a clinical evaluation only. However, based on objective diagnoses of deep vein thrombosis (DVT) and pulmonary embolism (PE), studies report an incidence of VTE of between 0.6 and 1.3 cases per 1000 deliveries. This amounts to a 5–10 times higher rate than that observed in nonpregnant women [2].

According to the pregnancy-related mortality surveillance performed by the CDC between 1991 and 1999, PE was the leading cause (in 20%) of pregnancy-related deaths, which was higher than other pregnancy-related complications, such as hemorrhage, infections, and pregnancy-induced hypertension [3].

The risk of thrombosis during pregnancy is attributed to homeostatic changes that occur during this period. During normal pregnancy, the concentrations of the clotting factors fibrinogen, VII, VIII, von Willebrand factor, IX, X, and XII are all increased, resulting in a hypercoagulable state, which exposes pregnant women to an increased risk of thrombosis [4].

Moreover, the mechanical obstruction by the growing uterus compromises venous outflow and subsequently increases the susceptibility of pregnant and postpartum women for developing thromboembolisms [5]. Moreover, pregnancy combined with either heritable or acquired forms of thrombophilia constitutes a cumulative risk of thrombosis [6].

The present study was conducted in a single hospital in Riyadh to address the lack of research data on pregnancy-induced thrombosis in Saudi Arabia, analyze the circumstances surrounding cases of pregnancy-induced VTE (DVT and PE), identify potential factors triggering thrombosis (i.e., thrombophilia, obesity, age, parity, and family history), determine the sites and clinical presentations of VTE, analyze its diagnostic methods, elucidate effects of initial- and long-term management, and assess recurrence rates and mortality of VTE among pregnant Saudi women.

## 2. Materials and Methods

### 2.1. Study Design

A retrospective chart review was conducted for all objectively confirmed VTE patients (i.e., those with DVT, PE, or both), occurring during pregnancies or postpartum period from January 2010 to November 2015, using the thrombosis clinic registry at King Fahad Medical City, Riyadh, Saudi Arabia.

All patients who experienced one or more episodes of objectively confirmed VTE during pregnancy or postpartum period were included in this study. Patients with unusual site thrombosis (i.e., any thrombosis other than DVT or PE) and those with either missing medical records or with normal outcomes of diagnostic imaging were excluded.

### 2.2. Data Collection

The following demographic data were collected for analysis: age, weight, height, body mass index (BMI), family history of VTE, previous history of oral contraceptive use, and the pregnancy trimester at the time of VTE diagnosis. Patients were categorized based on their pregnancy status (antenatal or postnatal), VTE, and trimester of pregnancy.

Depending on their VTE diagnosis, patients were allocated to one of three cohort groups (i.e., DVT, PE, and DVT progressed to PE), and their DVT site was classified as right/upper or lower limb or as left/upper or lower limb). Diagnoses were objectively confirmed by Doppler ultrasound in cases with DVT and with a ventilation-perfusion scan or computed tomography pulmonary angiography scan in cases with PE.

Risk factors underlying the development of VTE were determined using the risk assessment tool of the Royal College of Obstetricians and Gynecologist (RCOG) [7].

Information regarding both acute/initial and long-term treatment and about the outcomes, e.g., VTE recurrence or maternal mortality, were extracted from the patients' records.

### 2.3. Ethical Approval

The study was approved by the Institutional Review Board of King Fahad Medical City, Riyadh, Saudi Arabia (Protocol # RC15-360). The study was conducted according to the recommendations of the International Conference on Harmonization for Good Clinical Practice (ICH-GCP).

### 2.4. Statistical Analysis

Data were entered and analyzed using the SPSS software (version 19; SPSS Inc., Chicago, IL, USA). The analysis consisted of descriptive group parameters. Continuous variables were processed as mean ± standard deviation. Categorical variables were analyzed as frequencies with corresponding percentages within the different categories.

## 3. Results

During the study period, 800 VTE cases were identified. Out of them, 180 patients were diagnosed with pregnancy-induced VTE (135 (75%) patients developed DVT, 30 (16.7%) patients developed PE, and 15 (8.3%) developed DVT that progressed to PE)).

Patient demographic data revealed a mean age of 29.67 ± 5.9 years and a BMI of 31.76 ± 6.4 kg/cm2. VTE cases were almost equally distributed, with a slight surge toward the first and third trimester (33.8% and 32.4%, respectively; Table 1). Overall, 60% (*n* = 109) of the VTE cases occurred during the postpartum period, whereas 40% (*n* = 71) occurred during pregnancy (antenatal period).

### 3.1. DVT Sites and Clinical Presentations of VTE

Regarding the DVT sites, our results showed that among the 150 patients with DVT, the left leg was involved in 116 (77.4%) patients in whom the proximal site was the dominant site of involvement. Right leg DVT was observed in 15.5% of patients.

The patients with VTE (*n* = 180) showed varying clinical presentations, among which the most common were lower leg pain, lower limb swelling, and entire leg swelling (57.2%, 54.4%, and 35.6% respectively); other clinical presentations observed are shown in Table 2.

### 3.2. Risk Factors of Pregnancy-Associated Thrombosis Based on RCOG Risk Assessment

Cesarean section was the topmost prevalent risk factor among study participants, which was observed in 86 (47.8%) patients, followed by obesity (73 (40.6%) patients), multiparty (>3 children; 58 (32.2%) patients), the presence of medical comorbidities (such as T2DM, gestational DM, and hypertension; 56 (31.1%) patients), age >35 years (53 (29.4%) patients), and family history (19.4% of patients).

Risk factors that were less frequent include surgical procedures (3 (1.7%) patients), dehydration or ovarian hyperstimulation syndrome (OHSS; 3 (1.7%) patients), systemic infection (4 (2.2%) patients), preeclampsia (8 (4.4%) patients), and postpartum hemorrhage (PPH) or blood transfusion (8 (4.4%) patients; Figure 1).

OHSS: ovarian hyperstimulation syndrome; PPH: postpartum hemorrhage; VTE: venous thromboembolism; APLS: antiphospholipid syndrome; ART: assisted reproductive technologies; BMI: body mass index; C/S: cesarean section.

### 3.3. Diagnosis of Thrombophilia

Thrombophilia workup showed that 31 (17%) patients had thrombophilic abnormalities. The most common type was antiphospholipid syndrome (APLS; 14 (8%) patients), followed by protein S deficiency (12 (7%) patients). Other thrombophilic abnormalities included the presence of the factor V Leiden (FVL) or prothrombin gene mutation G20210A and protein C deficiency. All thrombophilia investigations were performed after treatment completion and after 6 weeks of delivery (Table 3).

### 3.4. Treatment and Outcomes

Among the antenatal patients (*n* = 71), most patients (67 (94.4%)) received low molecular weight heparin (LMWH), whereas 4 (5.6%) patients received unfractionated heparin (UFH). Among those who received LMWH, almost all patients (65 out of 67) received enoxaparin. The remaining two patients experienced enoxaparin allergy and received tinzaparin instead.

Among the postpartum patients (*n* = 109), similarly to pregnant patients, LMWH was used most often, i.e., in 93.5% of the patients, as initial treatment. Again, enoxaparin was administered to most patients (93.5%) and tinzaparin (2%) only to those with enoxaparin allergy. The UFH was used in 4.6% of the patients, while two patients (2.0%) received the factor Xa inhibitor rivaroxaban as initial treatment. Further, treatment regimen varied between oral anticoagulants and subcutaneous heparin: 34% (*n* = 61) of patients continued enoxaparin throughout the entire treatment course, 1% (*n* = 2) continued receiving tinzaparin, 48% (*n* = 86) were prescribed vitamin K antagonists (VKA; warfarin), and 17% (*n* = 31) received Factor Xa inhibitors (rivaroxaban) (Table 4).

The treatment duration was 3 months for 20.5% of the patients and 6 months for 43.0%. It further extended in 36.4% of the patients who had recurrent VTE or thrombophilic abnormalities.

Further, 2 maternal (1.1%) deaths occurred in the study cohort. There were 20 (11.1%) recurrences of VTE episodes, mostly in the form of DVT 15 (75%), PE 2 (10%), both DVT and PE 2 (10%) and CVT 1 (5%) (Figure 2).

In patients with recurrent VTE, pregnancy was the most observed provoking factor (55%, *n* = 11) followed by surgery and hospitalization (10% and 5%, respectively). Moreover, 6 cases experienced recurrent unprovoked VTE (i.e., not associated with an environmental risk factor), of which 3 had thrombophilia.

## 4. Discussion

The present study revealed that the frequency of pregnancy-associated thrombosis was greater during the postnatal than during the antenatal period (i.e., 60% vs. 40%, respectively). Moreover, our results revealed that cesarean section was the most prevalent risk factor among study participants, followed by obesity and multiparty. The most common clinical presentations were lower leg pain and lower limb swelling. Further, our results showed that approximately 11% of the participants had recurrences of VTE episodes, and maternal mortality occurred in 2 (1.1%) cases.

The observed increase in thrombosis risk among postpartum women agrees with the existing literature; a meta-analysis conducted to contrast the risk among these two groups estimated that the relative risk among 100 DVT events was 0.23 per day during pregnancy, against 0.83 per day during the postpartum period [7]. The MEGA study, a case-control study, found a five-fold increased risk of venous thrombosis during pregnancy and a 60-fold increase in the postpartum period, which could be attributed to either the mode of delivery, postnatal infections or level of immobility [1].

We found that the frequencies of thrombosis during the various pregnancy trimesters were roughly equal, with slight elevations seen in the first and third trimester (33.3% and 31.9% respectively); the RIETE, an ongoing Spanish registry of patients with VTE reported a similar incidence during the different trimesters, with higher overall levels (first and third trimester: 40% and 42%, respectively) [8].

In our study, the patients developed DVT more often than PE (25% vs. 75%), which is consistent with the results of a previous study [8]. For example, the RIETE registry reported that among pregnant and postpartum patients with VTE, 81% developed DVT, while only 18% of these patients developed PE [8].

Our results show that the vast majority of DVT cases occurred in the left leg, with the proximal site affected mainly. Similar findings were reported in a systematic review of the anatomical distribution of DVT in pregnancy. It was found that 88% of cases with DVT occurred in the left leg and that 71% were restricted to the proximal veins, without the involvement of the calf veins. The authors explained these findings as resulting from a May–Thurner-like syndrome, in which the left iliac vein is compressed by the gravid uterus in the area, where it crosses the right iliac artery. They suspected that this syndrome had a vital role in the increased incidence of iliofemoral DVT in late pregnancy [9].

The risk profile analysis of our patients revealed that obesity was the most prevalent risk factor, followed by multiparity. These findings are consistent with those from a large cross-sectional study in which obesity was manifest in 76% of the examined VTE cases, and multiparity was the second most prevalent risk factor observed in 33% of patients [10]. In another case-control study conducted among Sudanese pregnant and postpartum patients with VTE, it was found that family history, followed by multiparity and cesarean section delivery was the most significant risk factors (ORs: 7.4, 2.2, and 2, respectively) [11].

Other risk factors that have traditionally been linked to pregnancy-induced thrombosis in the literature [12], were also observed in our study, i.e., the history of thrombosis, multiple gestation, medical comorbidities, immobility, thrombophilia, and antiphospholipid syndrome.

Nearly half of the postnatal thrombosis cases had gone through a cesarean delivery, and many studies support the notion that cesarean section is associated with a doubled risk of thrombosis compared to vaginal delivery (OR = 2) [11, 12].

Seventeen percent (*n* = 31) of patients had either acquired or hereditary thrombophilia. Compared to the general population, thrombophilic abnormalities were increased 51.8-fold among individuals with hereditary thrombophilia [12].

The distribution of thrombophilic patterns in our study participants shows protein S deficiency to be the most common form of hereditary thrombophilia, while FV and protein C are the least common forms. This was in line with a study in the Saudi population, in which protein S deficiency was the most dominant form of thrombophilia (14.5%), whereas prothrombin gene mutations and FVL mutations were the least common cause for thrombophilia (in 1.1% and 0.5% of patients, respectively) [13]. However, this pattern of results stands in contrast with Western studies, in which the FVL mutation was shown to be the most prevalent pattern of thrombophilia [6, 14].

The mainstay of initial treatment for both pregnant and postpartum patients was enoxaparin, which is compatible with the American College of Chest Physicians and RCOG latest recommendations on VTE management in pregnancy and postpartum [15, 16]. One of the largest systematic reviews of LMWH use during pregnancy in which most of the included patients received enoxaparin both for treatment and prophylaxis (60% and 44%, respectively) concluded that LMWH is a safe and effective treatment or prophylactic for thrombosis in pregnancy [17].

Patients in their postpartum period continued to receive LMWH or were switched to oral VKA for least 6 weeks postnatal or total duration of treatment of 3 months' regardless of whether VTE occurred during pregnancy or the postpartum period, which is congruent with RCOG 2015 guidelines on the management of VTE in pregnancy [16].

The risk of recurrence after the first episode of pregnancy-associated thrombosis was 11%. Of these recurrences, 6.1% of the recurrences occurred during pregnancy, whereas 2% occurred in the presence of other transient provoking factors, and 3% developed recurrent unprovoked VTE, figures that are similar to earlier reports. For example, a systematic review of randomized trials examining the risk of recurrence VTE in patients with the first episode of symptomatic VTE provoked by a transient risk found a recurrence rate of 3.3% for all patients with a transient risk factor, of 0.7% in patients with surgical risk factors, of 4.2% in those with nonsurgical risk factors and, finally, of 7.4% after unprovoked VTE [18].

The mortality observed in our study was almost 1%, which is quite comparable to what has been reported, such as a recent meta-analysis of the epidemiology of VTE among pregnant women, which included 20 studies and found an overall mortality of 0.65% [19].

Our results can be a guide to policymakers to include VTE prevention among pregnant women in maternal and child healthcare programs, which can lead to the averting the morbidity associated with this disease on women's health and pregnancy outcomes as well as its associated mortality. Moreover, there is a need to develop educational programs to enhance the knowledge of the healthcare providers in handling VTE in pregnant women.

Our results will be a base for future research and contribute to developing and optimizing strategies to prevent and treat VTE in pregnant women. However, larger studies with randomized design and control groups are required to confirm and expand the results of our study and to understand risk factors for VTE and their possible countermeasures.

This is one of few studies conducted in the Kingdom of Saudi Arabia and is significant as it represents a database to determine the risk factors, laboratory profile, radiological imaging, and outcomes of management of pregnancy-related VTE at one of the most reputable tertiary healthcare institutions in Saudi Arabia.

A critical limitation of our study was the absence of a control group to compare and contrast the risk factors found in VTE patients. Moreover, the lack of prepregnancy BMI data was another limitation. It might have been more accurate to estimate the true effect of obesity from patients' baseline weight before pregnancy. Further, the study was conducted at a signal tertiary care hospital, which hinders the generalizability of the findings.

## 5. Conclusion

In the present study, pregnancy was the most frequently observed provoking factor in VTE, exceeding other transient risk factors such as surgery, hospitalization, and oral contraceptive use.

Also, an increased risk of VTE occurred in the postpartum period relative to that during pregnancy. Accordingly, we believe that all pregnant women should undergo a formal, written risk assessment of factors for VTE during the antenatal and perinatal period. Also, measures for VTE prophylaxis in patients with a history of VTE deserve special attention.

## Figures and Tables

**Figure 1:** Risk factors distribution among patients based on RCOG risk assessment.

**Figure 2:** Sites of VTE involvement in patients with VTE recurrence.

**Table 1:** Study participants' demographic data.

Variable		
Mean age (±SD) (years)	29.67 (±5.99)	
Mean body mass index (±SD)	31.76 (±6.48)	
Pregnancy status		
Antenatal	71	40%
Postpartum	109	60%
Pregnancy trimester		
1^st^ trimester	24	33.8%
2^nd^ trimester	18	25.3%
3^rd^ trimester	23	32.4%
Unknown trimester	6	8.5%
Family history		
Yes	35	19.4%

Data are presented as number and percentage or mean and standard deviation (SD).

**Table 2:** Clinical presentations of VTE (DVT and PE) and distribution of DVT site involvement in patients.

	*n*	%
DVT site (*n* = 150)		
Left leg DVT	116	77.4
Right leg DVT	23	15.3
Bilateral DVT	8	5.3
Upper limbs	3	2.0
Clinical presentations of VTE (*n* = 180)		
Lower leg pain	103	57.2
Lower limb swelling	98	54.4
Entire leg swelling	64	35.6
Shortness of breath	37	20.6
Chest pain	36	20.2
Calf swelling >3 cm	23	12.8
Localized tenderness	16	8.9
Pitting edema	10	5.6

**Table 3:** Distribution of thrombophilia types among patients.

Thrombophilic abnormalities	*n*	%
APLS	14	8.0
Protein S deficiency	12	7.0
Factor V Leiden mutation	2	1.0
Prothrombin gene mutation G20210A	2	1.0
Protein C deficiency	1	0.5

**Table 4:** Initial and maintenance treatment regimen in postpartum patients.

	*n* (%)
Initial treatment	
Enoxaparin	99 (93.5)
Tinzaparin	2 (2.0)
UFH	5 (4.6)
Rivaroxaban	2 (2.0)
Maintenance treatment	
Enoxaparin	61 (34.0)
Tinzaparin	2 (1.0)
Warfarin	86 (48)
Rivaroxaban	31 (17)

## Data Availability

The data are available with the corresponding author.
